The article "Fundus-Vascular Responses to Color Deviation Caused by Non-Oxidative Blue Filtering" was retracted in 2023. Reasons: signs of a paper mill; compromised peer review; unreliable results or conclusions.

# Fundus-Vascular Responses to Color Deviation Caused by Non-Oxidative Blue Filtering

**DOI:** 10.1155/2022/9592009

**Published:** 2022-10-12

**Authors:** Jianqi Cai, Wentao Hao, Shanshan Zeng, Junkai Li, Ya Guo, Kai Tan, Yongyin Kang, Yitao Huang, Yue Zhang, Thebano Santos, Cheng Qian, Aiqin Luo

**Affiliations:** ^1^School of Life Science, Beijing Institute of Technology, Beijing 100081, China; ^2^Lab of Visual Health and Safety Protection, China National Institute of Standardization, Beijing 100191, China; ^3^Beijing Yangming Zhidao Photoelectric Science and Technology Co., Ltd, Beijing 100102, China; ^4^Hangzhou Innovei Technology Co., Ltd, Hangzhou 311199, China; ^5^Guangzhou Shirui Electronics Co., Ltd, Guangzhou 510663, China; ^6^Najing Technology Co., Ltd, Hangzhou 310052, China; ^7^Center of Information Technology “Renato Archer” (CTI), Ministry of Science Technology Innovations and Communications, Brazil; ^8^School of Reliability and Systems Engineering, Beihang University, Beijing 100191, China

## Abstract

**Aims:**

Short-wavelength blue light damaged retina by the oxidative stress in the retinal pigment epithelial (RPE) cells. Filtering blue light from screen could reduce blue hazard, whereas it inevitably altered color-gamut coverage and color-deviation level. Although abnormal fundus-vascular density (FVD) sometimes indicated fundus disease, few researchers noticed its responses to the variation of color-gamut coverage and color-deviation level.

**Methods:**

In this study, we performed cellular experiments and analyzed the RPE cell viabilities (CVs) in spectrums with different blue (455-475 nm) ratios to describe the corresponding oxidative-stress levels. Further, we investigated the effects of color-gamut and deviation on FVD variations during the screen-watching task using human factor experiments with 30 participants (university students, including 17 males and 13 females, 21 to 30 years old).

**Results:**

RPE CVs were similar in different spectrums, implying that non-oxidative blue filtering hardly contributed to CV improvement. Color-deviation level seems to induce more significant effects on the visual function compared to color-gamut coverage, and MTF and FVD presents similar variation trends during the visual task.

**Conclusion:**

Oxidative-free blue filtering contributed little to decrease retinal oxidative stress yet caused color-deviation increase, which caused significant FVD reduction.

## 1. Introduction

Short-wavelength blue light threatens the RPE cells by increasing the risk of fundus diseases, comprising age-related macular degeneration (AMD) [1, 2], diabetic retinopathy (DR) [3, 4], idiopathic parafoveal telangiectasis (IPT) [5, 6], retinal vein occlusion (RVO) [7, 8], retinal artery occlusion (RAO) [9, 10], central serous chorioretinopathy (CSC) [11, 12], and polypoidal choroidal vasculopathy (PCV) [13, 14].

Although in display blue wavelength filtering reduced blue hazard, it caused other issues such as variations in color-deviation level and color-gamut coverage. Whether human eyes benefit from non-oxidative blue filtering remained unclear. Researchers have performed ergonomic studies to clarify the effects of display brightness [15–17] on visual and nonvisual effects [18–20], whereas they focused little on the fundus-vascular responses to different color-gamut coverages and color-deviation levels.

Generally, non-oxidative blue filtering is inevitably accompanied by several negative consequences, including complicated control circuits and algorithms [21], distorted display-input signals [22], and reduced color-deviation levels [23–25]. In this study, we measured FVD variations in different color-gamut coverages and color-deviation levels, which were caused by the non-oxidative blue filtering, during screen-watching tasks in experiences with human subjects. We also analyzed the correlation between FVD and MTF.

## 2. Materials and Methods

### 2.1. Light Environment

A light-emitting diode (LED) lamp fixed on a 2.1-m ceiling was used for lighting with the following characteristics: size of 90 cm × 90 cm and a correlated color temperature (CCT) of 5250 ± 250 K. The screen brightness was set to a value of 190 ± 10 cd/m^2^. Spectral power distributions (SPD) of the screen and the ceiling lamp are shown in Figure 1. To obtain all of the color features in this study, color corrections were performed using Truecolor Analyzer 2.6 software. A total of 15 screens presenting 15 color features (Table 1) were used.

### 2.2. Cellular Experiments

We carried out cellular experiments to investigate the effects of different spectrums. The retinal cells for this study were human ARPE-19 cells purchased from Procell Co. Ltd. We cultivated the ARPE-19 cells with the DMEM-F12 solution (10% fetal-calf serum) in the cell-culture incubator with 5% CO2. All the ARPE-19 cells were divided into three groups and cultivated in the screen with the three color-deviation levels shown in Table 1. The screens were set to the status of white balance, and the illuminance value was 400 lux.

For CV measurement, we performed cellular staining with the Trypan Blue and then analyzed the CV using the ThermoFisher Scientific Flow Cytometer instrument. CV data were automatically collected.

### 2.3. Human Factor Experiments

In this study, all 30 participants (university students, including 17 males and 13 females, 21 to 30 years old) provided written informed consent. All of the methods used were performed in accordance with the relevant guidelines and regulations. Participants were assessed to ensure that they had no oculopathies such as cataracts, heterotropia, or amblyopia. Based on the survey data from all participants, anisometropia levels were below 2.5 D, the intraocular pressure distribution ranged from 14 to 20, and the diopter distribution was as follows: 40% in the range −0.75–0.75 D and 60% in the range −1.00 D to −3.00 D. The corrected visual acuities were 0.8 (40%) and 1.0 (60%). All information on participants parameters are listed in Table 2.

We performed two visual tasks: a color-recognition task and a video-watching task. Both tasks were completed on 15 separate days, with a visual task and corresponding color status performed. Before the tasks, participants were asked to relax their eyes by looking into the distance for 20 mins. Next, the color-recognition task was administered. For this task, we used a 100-page document in portable document format (PDF) with 20 color options and a reference color box on each page. Each participant was asked to identify which color option was in the same color as the reference color box on each page. Each participant was given 20 mins to complete the color-recognition task. During this time, participants also performed the video-watching task. For the video-watching task, participants watched the movie “Angry Birds” (produced by Rovio Mobile and released on May 20th, 2016). The duration of the video-watching task was also 20 mins.

### 2.4. Human Ocular Measurements

We measured the FVD of each screen user prior to and following the screen-watching task. FVD was measured using an Optical Coherence Tomography Angiography (OCTA) instrument with RS-3000 equipment. The areas of the fovea vascular and avascular zones were automatically calculated for each participant and are shown in Figure 2 with the red and green colors representing the vascular area and the optic-disk area, respectively. We calculated FVD variations (*Δ*FVD) by subtracting the FVD data following the screen-watching task with the data collected prior to the task.

Each participant was asked to attach his or her forehead and chin to the specified location on the instrument and to look at the target on the screen binocularly under natural conditions. FVD data were collected automatically by the instrument. A training trial simulating the complete task content was run for each participant before data collection until the task was well understood.

We also collected the modulation-transfer function (MTF) as a supplementary piece of data. MTF was recorded using the NIDEK OPD Scan III, which collected data automatically. Likewise, all participants were allowed to blink during the measurement to avoid aggravation of ocular fatigue caused by extended interblink intervals. We calculated MTF variations (*Δ*MTF) by subtracting the final MTF (following the task) with the initial MTF (prior to the task).

To assess visual comfort levels by calculating the visual comfort (VICO) index, we measured the corneal-refractive power (KR), axial length (AL), ciliary accommodation (ACC), and high-order aberrations (HOAs): KR and AL values were measured using the NIDEK AL-Scan automatically. The NIDEK AR-1S instrument was used to collect the ACC automatically. For the HOA measurements, we used the NIDEK OPD Scan III to automatically collect the participants' data.

## 3. Results

### 3.1. CV Comparisons

We measured CVs in the color-deviation level of 0.9 < ΔE < 1.8, 1.8 < ΔE < 2.7, and 2.7 < ΔE < 3.6, and the results were 76.97%, 77.46%, and 77.15%, respectively (Figure 3). The CVs in the three color-deviation levels presented little differences, and the three corresponding spectrums were similar in their effects on CV. As the three spectrums were obtained by non-oxidative blue (455-475 nm) filtering, the non-oxidative blue light seemed to cause little damage to the retinal cells. Conversely, filtering the necessary blue light might induce color-deviation reduction.

### 3.2. *Δ*FVD Responses

We observed significant *Δ*FVD differences among the study participants (Table 3). Within the same color-deviation level, we did not identify any significant differences in *Δ*FVD values in different color-gamut coverages, implying that the variations of color-gamut coverage do not induce changes in *Δ*FVD. In contrast, we observed significant *Δ*FVD differences in different color-deviation levels (Table 4). In summary, differences in *Δ*FVD seemed to rely on the color-deviation level rather than the color-gamut coverage.

We observed bell-shaped distribution curves for *Δ*FVD values collected for various color-gamut coverages and color-deviation levels. Although changes in the color-gamut coverage hardly affected the locations of the bell-shaped curves, it caused their deformations. For each color-deviation level, the distribution curves grew more dispersive with the increase of the color-gamut coverage (Figures 4(a)–4(c)). The color-deviation level differed from the color-gamut coverage based on differential effects on FVD. With increased color-deviation levels, the bell-shaped distribution curves exhibited crests that were shifted toward higher values (Figures 4(d)–4(h)).

### 3.3. *Δ*MTF Responses

The *Δ*MTF data were similar to *Δ*FVD data in performance, as the color-gamut coverage variation altered the *Δ*MTF-distribution dispersity (Table 5, Figures 5(a)–5(c)) while the color-deviation-level variation caused the bell-shaped-curve's shift (Table 6, Figures 5(d)–5(h)). Compared to the color-gamut, the color-deviation level had a more significant effect on *Δ*MTF.

## 4. Discussion

### 4.1. *Δ*FVD-*Δ*MTF Correlation

During the screen-watching tasks, we found that the participants' ocular responses depended on both the color-deviation level and the color-gamut coverage. The *Δ*FVD and *Δ*MTF presented similar variation regularities, with their distribution curves deformed to be more dispersive with increases in color-gamut coverage and shifting toward higher values with a larger color-deviation level. The similar performances observed corresponded with their possible correlation, which was confirmed by correlation analysis using SPSS 20.0 software (Table 7). The correlation was significant for each color deviation and each type of color-gamut coverage. The MTF determines the spatial distribution of photos in photoreceptors, which attach to retinal vessels. The RVA describes blood circulation in retinal vessels. In our study, the *Δ*FVD-*Δ*MTF correlation indicated that retinal vessel circulation might vary with photoreceptor-activation distribution.

### 4.2. VICO Mapping

We used the VICO index to determine the effects of each color-deviation and color-gamut coverage on ocular fatigue. With a ΔE < 2.7, increased color-gamut coverage led to a decreased VICO. Furthermore, a color-gamut coverage of 82% NTSC was an inflection point that divided the VICO curve into different-slope parts (Figure 6). With an ΔE > 2.7, however, the VICO index did not change with the color-gamut coverage.

In this study, there were 15 combinations of color-deviation and color-gamut coverage (Table 2). By designating the color-gamut coverage as the horizontal coordinate and the color deviation as the vertical coordinate, we could graph all 15 combinations in a two-dimensional coordinate system as 15 dots, corresponding to 15 VICO values. Since the color-deviation and color-gamut coverage variations contributed to VICO values continuously, we simulated the VICO value for each dot in the two-dimensional coordinates (with a color-gamut range from 70% to 95% NTSC, and a color-deviation range from 1.5 to 5.5) using the Newton interpolation method (Figure 6). The VICO heat map showed that the color distribution contributed more significantly to VICO than the color-gamut coverage, and also showed that color-deviation modulated color-gamut coverage's effects on VICO. In the heat map, the yellow color is likely a boundary whose shape highlights the color-gamut coverage at 82% as the inflection point.

## 5. Conclusion

In this study, we analyzed fundus-vascular responses to color-deviation reduction caused by non-oxidative blue filtering. Variations in FVD were used to indicate fundus-vascular responses. Our results showed that color-gamut coverage variations caused altered dispersions in the distribution curves for *Δ*FVD and *Δ*MTF, while color-deviation changes induced distribution's curve shifts. We also discovered that ocular comfort relied on color deviation more than color-gamut coverage by VICO heat map, since the color transition was more rapid along the color-deviation- coordinate axis. Specifically, a color deviation of 2.7 seemed to be a VICO heat map boundary. Increased color-gamut coverage caused a reduction in VICO when ΔE < 2.7 and no longer induced VICO variation when ΔE > 2.7. As *Δ*MTF and *Δ*FVD were significantly correlated, we inferred that retinal-photon distribution determined the fundus-vascular activities in certain paths. Our findings showed that non-oxidative blue light did not damage retina; instead, it was necessary for display to decrease the reduction of fundus-vascular function. In display technology research and development, the role of non-oxidative blue wavelength is indispensable to limit the color-deviation increase and benefit visual function.

## Figures and Tables

**Figure 1:** Spectral power distributions (SPDs) of the screen and ceiling lamp.

**Figure 2:** FVD results. The red number represents the vascular area and the green number represents the optic-disk area.

**Figure 3:** CVs in different spectrums corresponding to the color-deviation level of 0.9 < ΔE < 1.8, 1.8 < ΔE < 2.7, and 2.7 < ΔE < 3.6, respectively.

**Figure 4:** *Δ*FVD-distribution curves induced by various color-gamut coverages in the range of (a) 0.9 < E < 1.8, (b) 1.8 < E < 2.7, and (c) 2.7 < E < 3.6, and caused by different color-deviation levels in (d) 95%, (e) 89%, (f) 82%, (g) 77%, and (h) 71%.

**Figure 5:** *Δ*MTF-distribution curves caused by various color-gamut coverages in the range of (a) 0.9 < E < 1.8, (b) 1.8 < E < 2.7, and (c) 2.7 < E < 3.6 and caused by different color-deviation levels in (d) 95%, (e) 89%, (f) 82%, (g) 77%, and (h) 71%.

**Figure 6:** VICO heat map in the two-dimensional coordinates of color-deviation and color-gamut coverage.

**Table 1:** Color features of screens used in the study.

Screen ID	Color-gamut (% NTSC)	Color-deviation (*Δ*E) level
1	71%	0.9 < ΔE < 1.8
2	77%	
3	82%	
4	89%	
5	95%	

6	71%	1.8 < ΔE < 2.7
7	77%	
8	82%	
9	89%	
10	95%	

11	71%	2.7 < ΔE < 3.6
12	77%	
13	82%	
14	89%	
15	95%	

**Table 2:** Test sample information based on participants visual task experiments.

Participant item	Distribution
Anisometropia	(i) <2.5 D
Intraocular pressure	(i) 14-20
Diopter	(i) − 0.75 D to 0.75 D: 40%
	(ii) − 1.00 D to − 3.00 D: 60%
Corrected visual acuity	(i) 0.8: 40%
	(ii) 1.0: 60%
Male-female ratio	(i) Males: 17
	(ii) Females: 13

**Table 3:** Comparisons of *Δ*FVD between the adjacent color-gamut coverage pairs in multiple color-deviation levels; *t* represents Student's *t*-test value, and *P* represents significance probability; ^∗^*P* < 0.05 and ^∗∗^*P* < 0.01.

Color-deviation Level	Color-gamut Coverages	*t*	*P*
0.9 < ΔE < 1.8	95% vs 89%	− 0.589	0.561
	95% vs 82%	− 1.132	0.267
	95% vs 77%	− 0.659	0.515
	95% vs 71%	− 1.410	0.169
	89% vs 82%	− 0.553	0.585
	89% vs 77%	− 0.181	0.858
	89% vs 71%	− 1.072	0.293
	82% vs 77%	0.451	0.655
	82% vs 71%	− 0.211	0.834
	77% vs 71%	− 0.680	0.502

1.8 < ΔE < 2.7	95% vs 89%	0.172	0.864
	95% vs 82%	− 0.421	0.677
	95% vs 77%	− 0.247	0.807
	95% vs 71%	0.041	0.967
	89% vs 82%	− 0.652	0.520
	89% vs 77%	− 0.403	0.690
	89% vs 71%	− 0.115	0.910
	82% vs 77%	0.230	0.820
	82% vs 71%	0.545	0.590
	77% vs 71%	0.390	0.700

2.7 < ΔE < 3.6	95% vs 89%	0.41	0.685
	95% vs 82%	0.342	0.735
	95% vs 77%	− 0.519	0.608
	95% vs 71%	− 0.724	0.475
	89% vs 82%	0	1
	89% vs 77%	− 0.970	0.340
	89% vs 71%	− 1.292	0.207
	82% vs 77%	− 0.798	0.432
	82% vs 71%	− 1.407	0.171
	77% vs 71%	− 0.224	0.824

**Table 4:** Comparisons of *Δ*FVD between the adjacent color-deviation level pairs in multiple color-gamut coverages; *t* represents Student's *t*-test value, and *P* represents significance probability; ^∗^*P* < 0.05 and ^∗∗^*P* < 0.01.

Color-gamut Coverage	Color-deviation Levels	*t*	*P*
95%	1.5 vs 2.3^∗^	2.503	0.018
	2.3 vs 3.3^∗∗^	4.343	0.001
89%	1.5 vs 2.3^∗∗^	3.452	0.002
	2.3 vs 3.3^∗∗^	4.611	0.001
82%	1.5 vs 2.4^∗∗^	3.452	0.002
	2.4 vs 3.3^∗∗^	6.413	0.001
77%	1.6 vs 2.4^∗∗^	3.417	0.002
	2.4 vs 3.3^∗∗^	5.541	0.001
71%	1.6 vs 2.4^∗∗^	4.019	0.001
	2.4 vs 3.4^∗∗^	3.983	0.001

**Table 5:** Comparing *Δ*MTF between the adjacent color-gamut coverage pairs in multiple color-deviation levels; *t* represents Student's *t*-test value, and *P* represents significance probability; ^∗^*P* < 0.05 and ^∗∗^*P* < 0.01.

Color-deviation Level	Color-gamut Coverages	*t*	*P*
0.9 < ΔE < 1.8	95% vs 89%	− 0.367	0.717
	95% vs 82%	− 0.711	0.483
	95% vs 77%^∗∗^	− 3.456	0.002
	95% vs 71%^∗∗^	− 3.269	0.003
	89% vs 82%	− 0.317	0.754
	89% vs 77%^∗^	− 2.683	0.012
	89% vs 71%^∗^	− 2.247	0.033
	82% vs 77%^∗^	− 2.766	0.01
	82% vs 71%^∗^	− 2.506	0.018
	77% vs 71%	0.268	0.791

1.8 < ΔE < 2.7	95% vs 89%	− 1.204	0.238
	95% vs 82%	0.593	0.558
	95% vs 77%	− 0.258	0.798
	95% vs 71%	0.162	0.873
	89% vs 82%	1.978	0.058
	89% vs 77%	0.772	0.446
	89% vs 71%	1.264	0.217
	82% vs 77%	− 1.431	0.164
	82% vs 71%	− 0.548	0.588
	77% vs 71%	0.708	0.458

2.7 < ΔE < 3.6	95% vs 89%	0	1
	95% vs 82%	− 0.187	0.853
	95% vs 77%	1.714	0.098
	95% vs 71%^∗^	2.711	0.011
	89% vs 82%	− 0.207	0.837
	89% vs 77%	1.791	0.084
	89% vs 71%^∗∗^	2.823	0.009
	82% vs 77%	1.622	0.116
	82% vs 71%∗	2.295	0.029
	77% vs 71%	1.409	0.170

**Table 6:** Comparing *Δ*FVD between the adjacent color-deviation-level pairs in multiple color-gamut coverages; *t* represents Student's *t*-test value, and *P* represents significance probability; ^∗^*P* < 0.05 and ^∗∗^*P* < 0.01.

Color-gamut Coverage	Color-deviation Levels	*t*	*P*
95%	1.5 vs 2.3^∗∗^	6.453	0.001
	2.3 vs 3.3^∗∗^	7.973	0.001
89%	1.5 vs 2.3^∗∗^	4.667	0.001
	2.3 vs 3.3^∗∗^	11.829	0.001
82%	1.5 vs 2.4^∗∗^	10.029	0.001
	2.4 vs 3.3^∗∗^	6.696	0.001
77%	1.6 vs 2.4^∗∗^	8.865	0.001
	2.4 vs 3.3^∗∗^	11.258	0.001
71%	1.6 vs 2.4^∗∗^	12.339	0.001
	2.4 vs 3.4^∗∗^	11.333	0.001

**Table 7:** Correlation between *Δ*FVD and *Δ*MTF with different color-gamut coverings and color-deviation levels; *t* represents Student's *t*-test value, and *P* represents significance probability; ^∗^*P* < 0.05 and ^∗∗^*P* < 0.01.

Color-deviation Level	Color-gamut Covering	Correlation coefficient	*P*
0.9 < ΔE < 1.8	71%^∗∗^	0.491	0.006
	77%^∗∗^	0.521	0.003
	82%^∗∗^	0.510	0.004
	89%^∗∗^	0.486	0.006
	95%^∗^	0.451	0.012

1.8 < ΔE < 2.7	71%^∗^	0.455	0.012
	77%^∗∗^	0.469	0.009
	82%^∗∗^	0.479	0.007
	89%^∗∗^	0.464	0.010
	95%	0.420	0.021

2.7 < ΔE < 3.6	71%^∗∗^	0.483	0.007
	77%^∗^	0.450	0.013
	82%^∗^	0.448	0.013
	89%^∗^	0.444	0.014
	95%^∗∗^	0.536	0.002

## Data Availability

The data that support the findings of this study are available from the corresponding authors upon reasonable request.
